The article "LncRNA NEAT1 promotes malignant phenotypes and TMZ resistance in glioblastoma stem cells by regulating let-7g-5p/MAP3K1 axis" was published in 2020. Journal: Biosci Rep.

# LncRNA NEAT1 promotes malignant phenotypes and TMZ resistance in glioblastoma stem cells by regulating let-7g-5p/MAP3K1 axis

**DOI:** 10.1042/BSR20201111

**Published:** 2020-10-30

**Authors:** Chang-Long Bi, Jin-Fang Liu, Ming-Yu Zhang, Song Lan, Zhuan-Yi Yang, Jia-Sheng Fang

**Affiliations:** Department of Neurosurgery, Xiangya Hospital, Central South University, Changsha 410008, Hunan Province, P.R. China

**Keywords:** Glioma stem cells, let-7g-5p, lncRNA, MAP3K1, NEAT1, Temozolomide

## Abstract

Glioblastoma multiforme (GBM) is one of the most malign brain tumors in adults. Temozolomide (TMZ) is an oral chemotherapy drug constituting the backbone of chemotherapy regimens utilized as first-line treatment of GBM. However, resistance to TMZ often leads to treatment failure. In the present study, we explored the expression and related mechanisms of nuclear enriched abundant transcript 1 (NEAT1) in glioma stem cells (GSCs). Quantitative real-time PCR (qRT-PCR) showed that NEAT1 was up-regulated in serum samples of GBM patients and GSCs isolated from U87, U251 cell lines. Functional experiments showed that NEAT1 knockdown restrained malignant behaviors of GSC, including proliferation, migration and invasion. Dual-luciferase assays identified let-7g-5p was a downstream target and negatively adjusted by NEAT1. Restoration of let-7g-5p impeded tumor progression by inhibiting proliferation, migration and invasion. Mitogen-activated protein kinase kinase kinase 1 (MAP3K1), as a direct target of let-7g-5p, was positively regulated by NEAT1 and involved to affect the regulation of NEAT1 on GSCs’ behaviors. In conclusion, our results suggested that NEAT1 promoted GSCs progression via NEAT1/let-7g-5p/MAP3K1 axis, which provided a depth insight into TMZ resistance mechanism.

## Introduction

As the most common primary intracranial tumor, glioblastoma multiforme (GBM) accounts for 40–50% of brain tumors [1]. The clinical symptoms of glioma are characterized by increased intracranial pressure and intracranial compression, with high morbidity, high recurrence rate, high mortality and poor cure rate [2–4]. Malignant gliomas have complex pathological mechanisms with high heterogeneity and plasticity, which brings great difficulty to treatment and diagnosis of disease [5,6]. At present, temozolomide (TMZ), as a representative drug of GBM treatment, has achieved significant curative effect in the treatment of GBM, especially in the GBM or anaplastic astrocytoma [7]. Unfortunately, a large proportion of patients are already resistant to TMZ, which has become a major barrier to GBM treatment [8–10]. Glioma stem cells (GSCs) are a small population of glioma cells, which become a major cause of disease recurrence and drug resistance generation due to the stemness such as self-renewal, unlimited proliferation and tumorigenicity [11]. Therefore, studies on the behaviors and related chemoresistance mechanisms of GSCs are of great significance for the search of new targets in the treatment of gliomas.

Long non-coding RNA (lncRNA) belongs to non-coding RNA, which have a length of more than 200 nucleotides [12]. Studies have shown that lncRNA play a vital role in many processes such as dose compensation effect, epigenetic regulation, cell cycle and cell differentiation regulation [13]. It was reported that lncRNA could maintain the stemness, self-renewal, proliferation and invasion capability of stem cells [14–17], but there are few studies on how lncRNA is involved in the regulation of chemoresistance in GSCs. Nuclear enriched abundant transcript 1 (NEAT1), a 4-kb lncRNA, is located in the nucleus and acts as proto-oncogenes in various cancers including glioma [18–20]. However, the action mechanism of NEAT1 in GSCs is not well illustrated and the effects between NEAT1 and TMZ resistance in GSCs is not reported by previous studies.

MicroRNAs (MiRNAs) also are a class of non-coding RNAs, engaged in the post-transcriptional regulation of genes [21]. Their abnormal expression or dysfunction often occurs in various diseases such as cardiovascular diseases, autoimmune diseases and tumors [21]. In tumor-related reports, miRNAs can be defined as tumor activators or tumor suppressors depending on the nature of the target genes [22]. Let-7g-5p was a member of let-7 family, which was confirmed significantly down-regulated in glioma patients [23]. High expression level of let-7g-5p was significantly associated with better prognosis of GBM patients [24]. However, the regulatory roles and underlying mechanism of let-7g-5p in GSCs are still lacking.

In the current study, we aimed to study the pathway of NEAT1-mediated regulation of GSCs behaviors and TMZ resistance. Hence, we examined the expression levels and biological functions of NEAT1, let-7g-5p and mitogen-activated protein kinase kinase kinase 1 (MAP3K1) in GBM patients or GSCs and further validated the molecular interactions. Finally, our results of the present study will provide a new insight into new therapeutic target and pathological mechanism research of GBM.

## Materials and methods

### Clinical sample collection

The peripheral blood samples of GBM patients (*n*=22) and normal volunteers (*n*=22) were collected in the Neurosurgery Department of Xiangya Hospital. Informed consent forms were signed by all participating patients, and the protocol was approved by the Ethics Committee of Xiangya Hospital of Centre South University. The blood samples were immediately used to prepare serum.

### Serum extraction

After collection of the peripheral blood samples, allow the blood to clot at room temperature for 30 min. The pellet was removed by centrifuging at 2000×***g*** for 10 min in a refrigerated centrifuge. After centrifugation, the liquid component (serum) was immediately transferred into a tube and the serum was maintained at 4°C while handling. Serum samples were stored at −80°C until use.

### RNA extraction and quantitative real-time PCR

All experiments were performed according to the manufacturer’s protocols. Total RNA from serum samples and tumor cells were extracted using TRIzol® reagent (Invitrogen, Thermo Fisher Scientific Inc). Cells or serum samples were lysed in TRIzol solution according to a proper proportion, and chloroform was added and mixed. Then the solution was centrifuged at 12000×***g***. The supernatant was transferred to a new tube, and then, an equivalent volume of isopropanol was added. After incubating for 20–30 min at 4°C, the mixture was centrifuged for 10 min at 12000×***g***. The supernatant was discarded and the pellet was washed with 75% ethanol. The pellet was resuspended in 20–50 µl of RNase-free water by pipetting up and down. Next, NanoDrop™ 2000 Spectrophotometers (Thermo Fisher Scientific, Inc.) were utilized to test RNA quality. Then the total RNA samples were used to synthesize cDNA by PrimeScript™ RT Reagent Kit (Takara, Dalian, China). Quantitative real-time PCR (qRT-PCR) was used to determine the expressions of NEAT1, let-7g-5p and MAP3K1 using SYBR® Green Real-Time PCR Master Mix (Thermo Fisher Scientific, Inc.) on ABI StepOne Plus™ Real-Time PCR System (Applied Biosystems, U.S.A.). Each sample was assessed in triplicate. *GAPDH* and *U6* were used as reference genes and primer sequence of tested genes were listed below:

GAPDH: forward 5′- CCATCTTCCAGGAGCGAGAT-3′;
GAPDH: reverse 5′-TGCTGATGATCTTGAGGCTG-3′;
U6: forward 5′-CTCGCTTCGGCAGCACA-3′;
U6: reverse: 5′-AACGCTTCACGAATTTGCGT-3′;
NEAT1: forward: 5′-ATGCCACAACGCAGATTGAT-3′;
NEAT1: reverse: 5′-CGAGAAACGCACAAGAAGG-3′;
let-7g-5p: forward: 5′-GAGTTCCTCCAGCGCTCCGT-3′;
let-7g-5p: reverse: 5′-GATGAGCAGGGTGACGCCAT-3′;
MAP3K1: forward: 5′-CAGAATCACACCACCCCGA-3′;
MAP3K1: reverse: 5′-CGGAGCATCACAAATAGCAGA-3′.

### Cell culture and CD133^+^ cell isolation

Human GBM cell lines (U87 and U251) and human embryonic kidney (HEK) 293T cells were acquired from the Chinese Academy of Medical Sciences (Beijing, China). The culture medium was Dulbecco’s Modified Eagle’s Medium (DMEM) with 10% fetal bovine serum (FBS, Gibco, Carlsbad, CA, U.S.A.). Cells were incubated at 37°C with 5% CO_2_.

For CD133^+^ cells isolation, U87 and U251 cells were suspended after addition of Fc receptor (FcR) reagents (Cat. BUF041B, AbD, Serotec) for blocking. Then, microbeads were added which were previously mixed with CD133 antibody (ab19892, Abcam, Cambridge, MA), and the mixture was incubated at 37°C for 1 h. After removing the magnetic beads, CD133^+^ cells were harvested as GSCs and cultured in Dulbecco's modified Eagle's medium and Ham's F12 (DMEM-F12) medium without serum (Invitrogen, U.S.A.) added with 10 ng/ml basic fibroblast growth factor (bFGF, Invitrogen, U.S.A.), 20 mg/ml epidermal growth factor (EGF, Invitrogen) and 2% B27 (Invitrogen, U.S.A.). The incubator was set to 37°C with 5% CO_2_.

### Sphere formation assay

CD133^+^ cells were dissociated into single cells with enzyme and transferred to 96-well plates in nonadherent conditions at optimal density (500–1000 cells). The medium mentioned above was used for culture. Half of the medium was renewed every 2 days, and the cells were then fixed with 4% formalin after 6 `days. The morphology of spheres was photographed under electron microscope.

### Flow cytometry assay

The cells isolated from spheres and U87 and U251 cells with CD133 magnetic beads were washed and incubated with PE-conjugated CD133 or CD44 antibody (Santa Cruz Biotechnology, U.S.A.). The dilution was prepared at 1:10 in phosphate-buffered saline (PBS)–bovine serum albumin (BSA) at 4°C for 30 min. In control group, cells were cultured with isotype IgG antibody. Cell counting analysis was performed using FACScan and FACSAria, respectively (BD Biosciences).

### Cell transfection

The short hairpin RNA (shRNA) of NEAT1 and its negative control (sh-NC), as well as let-7g-5p mimics, anti-let-7g-5p and their respective NC (mimics NC and anti-NC) were synthesized by Gene Pharma (Shanghai, China). The full sequence of NEAT1 and MAP3KA were cloned into pcDNA-3.1 vector (Thermo Fisher Scientific). Cell transfection was performed according to the protocol of Lipofectamine 2000 Reagent (Invitrogen, U.S.A.). In brief, Lipofectamine reagent and plasmids were diluted in Opti-MEM medium according to the prescribed ratio and incubated for 5 min at room temperature. Then, the diluted Lipofectamine reagent and plasmids were mixed at 1:1 ratio and incubated for 20 min at room temperature. Next, the mixture was added into cells and cultured for 48 h, then, the transfection efficiency was determined using qRT-PCR.

### Dual-luciferase reporter assays

NEAT1 and MAP3K1 3′-untranslated region (3′-UTR) sequences containing wild-type (WT) or mutation-type (MUT) binding site of let-7g-5p were amplified and integrated into pmirGLO vectors (Promega, Madison, WI, U.S.A.) and then transfected into HEK-293T cells using Lipofectamine 2000 Reagent. A dual-luciferase reporter assay kit (Promega) was utilized to evaluate the luciferase activity after transfecting with let-7g-5p mimics or mimics NC for 48 h.

### Cell viability assay

Cell proliferation was assessed through Cell Counting Kit-8 (CCK-8) assay (Beyotime Institute of Biotechnology, Jiangsu, China). Cells were put in a 96-well plate and cultured at 37°C for 48 h. Ten microliters of CCK-8 solution was added into each well and incubated at 37°C for 2 h; the absorbance at 450 nm was measured for cell viability assessment at 48 h (Figure 2A) or 0, 24, 48, 72 h (Figures 2C, 3D, 4E and 6B).

### Cell migration and invasion assays

Polyethylene terephthalate (PET)-based migration chambers and BD BioCoat Matrigel invasion chambers (BD Biosciences, Bedford, Massachusetts, U.S.A.) with a porosity of 8 μm were used for transwell cell migration and invasion assays. The same number of tumor cells (2 × 10^4^) in DMEM without serum were put on to the uncoated or Matrigel-coated filters of the upper chambers. DMEM/F12 with 15% FBS was added to the lower chamber. After 36–48 h of incubation, the cells on the surface of the filter were removed, the filter was fixed with 100% methanol and stained with Crystal Violet. The migration and invasion abilities of glioma cells were calculated with the mean number of cells in all fields of view and presented as the ratio of migrated and invaded cells to the initial cells. The experiment was performed three times independently.

### Western blot

Cells were collected and lysed in RIPA buffer containing protease inhibitors (Beyotime Institute of Biotechnology) to extract total protein. Equal protein (30 μg) was separated by 10% SDS/PAGE gel, and transferred to a PVDF membrane (Invitrogen, U.S.A.). Then followed by blocking with 5% skim milk powder in Tris Buffered Saline Tween (TBST). The membrane was then incubated with primary antibody including MAP3K1 (1:500, Rabbit polyclonal antibody, Abcam, Cambridge, MA, U.S.A.), N-cadherin (1:1000, Rabbit polyclonal antibody, Abcam, Cambridge, MA, U.S.A.), E-cadherin (1:1000, Rabbit polyclonal antibody, Abcam, Cambridge, MA, U.S.A.), GAPDH (1:2000, Rabbit monoclonal antibody, Cell Signaling Technology, Danvers, MA, U.S.A.) for 4°C overnight. Next, the membrane was washed using TBST every 5 min for three times, and then cultured with mouse anti-goat IgG secondary antibody (1:2000, monoclonal antibody, Santa Cruz Biotechnology, Santa Cruz, CA, U.S.A.) for room temperature at 2 h. After washing, the bands were imaged using Gel Imaging System (#1708370, Life Science), and band intensity was examined by ImageJ V1.8.0.

### Statistical analysis

Data were expressed as the mean ± SD. SPSS 13.0 software was used to analyze experiment data. Statistical significance was analyzed by Student’s *t* test or ANOVA for functional analysis. A statistical significance was defined at *P*<0.05.

## Results

### NEAT1 is up-regulated in GBM patients and GSCs

We collected the peripheral blood samples of GBM patients and normal volunteers to determine the expression of NEAT1 using qRT-PCR. As shown in Figure 1A, the expression level of NEAT1 was much higher in serum samples of GBM patients compared with that of healthy volunteers. It has been reported that aberrant NEAT1 could regulate the malignant progression of GSCs [18]. Therefore, we sought to examine the expression of NEAT1 in GSCs. First, CD133^+^ cells were isolated from U87 and U251 cell lines by CD133 magnetic beads, and FACS assay was conducted to detect the isolation efficiency. The results suggested that CD133^+^ cell approximately accounted for 4.34% of the total population in U87 cells and approximately accounted for 7.24% total population of U251 cells, whereas, after isolation, the CD133^+^ cell proportion approximately accounted for 87.35 and 92.46% of total cells, respectively (Figure 1B). Then, the CD133^+^ cells isolated from U87 and U251 cell lines were induced in stem cell medium and allowed to form cell spheres (Figure 1C). FACS detection showed that most cells of the spheres expressed stem cell antigen CD133 and CD44, indicating that the GSCs were successfully isolated and induced (Figure 1D). Finally, we collected CD133^+^/CD44^+^ and CD133^−^/CD44^−^ cells and labeled them as GSCs-U87/GSCs-U251 and non-GSCs-U87/non-GSCs-U251, respectively. qRT-PCR was performed to detect NEAT1 expression and the results indicated NEAT1 had a greater expression in GSCs cells compared with that in non-GSCs cells (Figure 1E). Collectively, the above results demonstrated that NEAT1 might be closely associated with the progression of GBM and GSCs’ behaviors.

**Figure 1:** NEAT1 is up-regulated in GBM patients and GSCs (**A**) Expression level of NEAT1 in the serum sample of normal volunteers and GBM patients using qRT-PCR. (**B**) FACS assay was performed to examine the CD133^+^ cell proportion in cells before and after the isolation of U87 and U251. (**C**) CD133^+^ U87 and CD133^+^ U251 glioma cells cultured in serum-free medium formed spheres. (**D**) Stem cell antigen markers on the surface of GSCs (CD133, CD44) were determined in single-cell spheres using FACS assay. (**E**) qRT-PCR was performed to detected the expression of NEAT1 in GSCs cells and non-GSCs. Data were expressed as the mean ± SD, *P<0.5, **P<0.01.

### Silencing NEAT1 enhanced the sensitivity of GSCs to TMZ and inhibited the malignant phenotypes

We investigated whether NEAT1 has effects on the sensitivity to TMZ and behaviors of GSCs. First, we detected the sensitivity of GSCs to TMZ by CCK-8 assay and screened the optimal TMZ concentration. The results demonstrated that GSCs had stronger resistance to TMZ compared with non-GSCs. However, with the increase in TMZ concentration, the survival rate of GSCs became lower correspondingly, and 400 μM TMZ had better inhibitory effect in GSCs (Figure 2A). Then, shRNA was utilized to knockdown the expression of NEAT1. The results of qPCR showed that NEAT1 expression level was significantly decreased after treatment with TMZ, and it was further inhibited by shRNA of NEAT1 (Figure 2B). Next, the impacts of down-regulating NEAT1 on the phenotypes of GSCs were further explored. The data of CCK-8 assay showed that knockdown of NEAT1 markedly enhanced the anti-proliferation effect of TMZ in GSCs (Figure 2C). Similarly, knockdown of NEAT1 further intensified the inhibitory roles of migration and invasion of GSCs mediated by TMZ (Figure 2D,E). Furthermore, Western blot also showed that down-regulation of NEAT1 obviously enhanced the promotion of E-cadherin level and the inhibition of N-cadherin level induced by TMZ treatment (Figure 2F). All these results indicated that knockdown of NEAT1 further enhanced the sensitivity of GSCs to TMZ, and inhibited the malignant phenotypes of GSCs.

**Figure 2:** Silencing NEAT1 enhanced the sensitivity of GSCs to TMZ and inhibited the malignant phenotypes (**A**) GSCs-U87/U251 and non-GSCs-U87/U251 cells were treated with different concentrations of TMZ, and then CCK-8 assay was performed to measure cell viability. (**B**) The expression level of NEAT1 was examined by qRT-PCR after treating with TMZ or TMZ+shNEAT1. (**C**) Cell proliferation capacity was detected by CCK-8 assay to test the effect of NEAT1 on to the TMZ resistance of GSCs. (**D,E**) The migration and invasion capacities of GSCs were quantified by transwell after treating TMZ alone or co-treating TMZ+shNEAT1. (**F**) Western blot assay was used to evaluate the protein levels of E-cadherin and N-cadherin in GSCs after treating TMZ alone or co-treating TMZ+shNEAT1. Data were presented as mean ± SD; *P<0.5, **P<0.01, ***P<0.001.

### Restoration of let-7g-5p decreased the TMZ resistance and malignant phenotypes of GSCs

Previous evidence have reported that overexpressing let-7g-5p worked as tumor suppressor in GBM, and was correlated with the glioblastoma (GB) stem cell phenotypes and TMZ resistance [23]. Here, we investigated the effects of let-7g-5p in GSCs. The results of qRT-PCR certified that let-7g-5p had lower expression in GBM patients compared with normal volunteers (Figure 3A). Consistently, let-7g-5p expression in GSCs was also significantly down-regulated than that in non-GSCs cells (Figure 3B). Next, the roles of let-7g-5p on GSCs malignant biological behaviors was explored. Figure 3C was described that the level of let-7g-5p observably increased after treating with TMZ, and co-treatment with let-7g-5p mimics further facilitated let-7g-5p expression. Cell proliferation assay implied that overexpressing let-7g-5p further enhanced the inhibition on cell viability mediated by TMZ treatment (Figure 3D). Likewise, overexpression of let-7g-5p further repressed the migration invasion phenotypes of GSCs on the basis of TMZ treatment (Figure 3E,F). The results of Western blot assay demonstrated that N-cadherin was further down-regulated, while E-cadherin was up-regulated when let-7g-5p was overexpressed in TMZ-treated GSCs, further confirming that let-7g-5p repressed the metastasis of GSCs (Figure 3G). Overall, it is concluded that up-regulation of let-7g-5p further enhanced the sensitivity of GSCs to TMZ and suppressed the proliferation and metastasis phenotypes of GSCs.

**Figure 3:** Restoration of let-7g-5p decreased the TMZ resistance and malignant phenotypes of GSCs (**A**) The expression level of let-7g-5p in the serum samples of normal volunteers and GBM patients were calculated by qRT-PCR. (**B**) The expression level of let-7g-5p in GSCs and non-GSCs were analyzed using qRT-PCR. (**C**) qRT-PCR was implied to detect the level of let-7g-5p after treating with TMZ alone or co-treating with TMZ and let-7g-5p mimics. (**D**) Cell viability was detected by CCK-8 assay to analysis the effect of let-7g-5p up-regulation on TMZ resistance of GSCs. (**E,F**) The migration and invasion of GSCs after treating with TMZ alone or co-treating with TMZ and let-7g-5p mimics were measured by transwell. (**G**) Western blot assay was used to evaluate the protein levels of E-cadherin and N-cadherin in GSCs after treating TMZ alone or co-treating TMZ+let-7g-5p mimics. Data were presented as mean ± SD; *P<0.5, **P<0.01, ***P<0.001.

### let-7g-5p negatively affected the functions of NEAT1

Next, we wanted to clarify the regulatory relationship between NEAT1 and let-7g-5p. Analysis of Starbase database indicated that there may be a potential binding site between NEAT1 and let-7g-5p (Figure 4A). We verified the predicted binding site of NEAT1 and let-7g-5p by dual luciferase reporter gene assay, which showed that transfection of let-7g-5p mimics obviously reduced the dual luciferase activity of NEAT1-WT transfected cells, whereas no effect was observed between NEAT1-MUT transfected cells (Figure 4B). Then, we evaluated the correlation between NEAT1 and let-7g-5p expression by qRT-PCR. As the results showed, overexpression of NEAT1 by transfection with pcDNA-NEAT1 plasmids significantly inhibited the expression of let-7g-5p, while silencing NEAT1 by transfection with shNEAT1 dramatically increased let-7g-5p expression (Figure 4C). Likewise, the negative correlation between NEAT1 and let-7g-5p in clinical samples was validated by Pearson analysis (Figure 4D). Taken together, we could conclude a targeted inhibition relationship between NEAT1 and let-7g-5p. Subsequently, CCK-8 assay results presented that knockdown of let-7g-5p partially reversed the inhibition of cell viability induced by NEAT1 silenced of TMZ-treated GSCs (Figure 4E). Similarly, silencing NEAT1 mediated the inhibition on migration and invasion of TMZ-treated GSCs were significantly weakened after let-7g-5p knockdown (Figure 4F,G). Likewise, the modulatory impacts of NEAT1 down-regulation on the levels of N-cadherin and E-cadherin in TMZ-treated GSCs were also diminished by let-7g-5p knockdown (Figure 4H). Accordingly, the above results indicated that let-7g-5p negatively affected the biological effects of NEAT1 by interacting with NEAT1.

**Figure 4:** let-7g-5p negatively affected the functions of NEAT1 (**A**) Bioinformatics method (Starbase) was used to predict the potential binding site between NEAT1 and let-7g-5p. (**B**) Dual-luciferase reporter assay was used to evaluate targeted relationship. (**C**) qRT-PCR was used to test the regulatory correlation between NEAT1 and let-7g-5p on expression level. (**D**) The expression correlation of NEAT1 and let-7g-5p in clinical samples was analyzed by Pearson analysis. (**E**) CCK-8 assay was used to explore that the effect of let-7g-5p down-regulation on NEAT1-mediated GSCs resistance to TMZ. (**F,G**) Transwell assay was performed to assess the roles of let-7g-5p down-regulation on the capacities of migration and invasion of GSCs on the basis of TMZ+shNEAT1 co-treatment. (**H**) Western blot assay was used to evaluate the roles of let-7g-5p down-regulation on the levels of E-cadherin and N-cadherin mediated by TMZ and shNEAT1 co-treatment. Data were presented as mean ± SD; *P<0.5, **P<0.01, ***P<0.001.

### NEAT1 increased the expression of MAP3K1 by sponging let-7g-5p

MAP3K1 was proved to be associated with the pathological manifestations and survival of glioma [9]. In current work, we explored the relationship of MAP3K1 and NEAT1/let-7g-5p axis. Bioinformatics tools (TargetScan database) forecasted an 8-bp potential binding site between MAP3K1 and let-7g-5p (Figure 5A). Dual luciferase reporter assays showed that transfection of let-7g-5p mimics significantly diminished the dual luciferase activity of MAP3K1-WT transfected cells, but had no effect on cells transfected with MAP3K1-MUT (Figure 5B), implying a direct targeting relationship between MAP3K1 and let-7g-5p. Followed qRT-PCR results showed that MAP3K1 expression was significantly reduced after overexpressing let-7g-5p, and notably increased by silencing let-7g-5p (Figure 5C). In clinical expression and correlation analysis also suggested that MAP3K1 was up-regulated and inversely associated with let-7g-5p, suggesting MAP3K1 was negatively regulated by let-7g-5p (Figure 5D,E). Moreover, a positive relationship was found in clinical samples between the expression of MAP3K1 and NEAT1 (Figure 5F). The data of western blot assay also described that the expression of MAP3K1 was significantly reduced by NEAT1 silence while this inhibitory effect was abolished by let-7g-5p down-regulation (Figure 5G). The above results pinpointed the MAP3K1 was positively regulated by NEAT1 through interacting with let-7g-5p.

**Figure 5:** NEAT1 increased the expression of MAP3K1 by sponging let-7g-5p (**A**) Bioinformatics method (TargetScan) was employed to predict the potential binding site between MAP3K1 and let-7g-5p. (**B**) Interaction relationship between let-7g-5p and MAP3K1 was assessed by dual-luciferase reporter assay. (**C**) qRT-PCR was used to test the regulatory correlation between MAP3K and let-7g-5p on expression level. (**D**) The expression level of MAP3K1 in serum samples of normal volunteers and GBM patients was calculated by qRT-PCR. (**E**) The expressive correlation of MAP3K1 and let-7g-5p in clinical samples was analyzed by Pearson analysis. (**F**) The clinical expressive correlation of NEAT1 and let-7g-5p in GBM patients was analyzed by Pearson analysis. (**G**) Western blot was implied to assess the regulatory role of NEAT1 on MAP3K1. Data were presented as mean ± SD; *P<0.5, **P<0.01, ***P<0.001.

### MAP3K1 involved the regulatory roles mediated by NEAT1/let-7g-5p axis in GSCs

Next, we probed whether MAP3K1 is involved in the regulation of GSC phenotypes by NEAT1/let-7g-5p axis. We first executed Western blot to test the level of MAP3K1 and the results showed that MAP3K1 level was markedly decreased by TMZ treatment, and it was further reduced by silencing NEAT1, whereas it was obviously elevated by pcDNA-MAP3K1 plasmids (Figure 6A). We performed a series of experiments to study the effect of overexpressing MAP3K1 on NEAT1-mediated GSCs’ phenotypes. Proliferation assay identified that overexpression of MAP3K1 significantly reversed the inhibition role on the proliferation of GSCs mediated by TMZ treatment and NEAT1 silencing (Figure 6B). Likewise, overexpressing MAP3K1 significantly reversed the roles of NEAT1 down-regulation on the inhibition of migration and invasion in TMZ-treated GSCs (Figure 6C,D). Furthermore, overexpression of MAP3K1 significantly increased N-cadherin level and decreased E-cadherin level (Figure 6E), suggesting the effects of NEAT1 down-regulation on TMZ resistance and phenotypes were markedly weakened by MAK3P1. Taken together, MAP3K1 participated in the regulatory network of NEAT1 on TMZ resistance and biological phenotypes of GSCs.

**Figure 6:** MAP3K1 involved the regulatory roles mediated by NEAT1/let-7g-5p axis in GSCs (**A**) Western blot was conducted to test the protein level of MAP3K1 in GSCs after co-transfection with shNEAT1 and pcDNA-MAP3K1. (**B**) Cell vability was detected by CCK-8 assay to assess the role of MAP3K1 overexpression on NEAT1-mediated TMZ resistance of GSCs. (**C,D**) Transwell was performed to evaluate the influence of MAP3K1 up-regulation on NEAT1-mediated cell migration and invasion induced. (**E**) Western blot assay was used to evaluate the protein levels of E-cadherin and N-cadherin after co-treatment with TMZ+shNEAT1+pcDNA-MAP3K1. Data were presented as mean ± SD; *P<0.5, **P<0.01, ***P<0.001.

## Discussion

GSCs are a niche of glioma cells which have the ability of self-renewal, promotion of angiogenesis and multidifferentiation [25]. Traditional treatment against glioma may be limited due to drug resistance, easy recurrence, rapid metastasis and invasion, which is partly triggered by the existence of GSCs [7]. Therefore, treatment targeting GSCs has become promising options for glioma therapy [2,26]. In the current study, we proposed a new molecule regulatory mechanism for lncRNA-mediated TMZ resistance in GSCs.

TMZ, an alkylatig agent, constitutes the first-line chemotherapy for glioblastoma and other tumors that significantly increases overall survival [8]. However, resistance against TMZ usually leads to GBM recurrence and treatment failure [9,10]. Therefore, it is demanding to better interpret the mechanisms involved in TMZ resistance. Increasing evidences indicate that lncRNA is one of the critical regulators in TMZ resistance of glioma. For instance, Li et al. confirmed that knockdown of LINC00174 reduced the chemoresistance of TMZ in GBM cells by regulating miR-138-5p/SRY-box transcription factor 9 (SOX9) axis [27]. Li et al. certified that lncRNA small nucleolar RNA host gene 15 (SNHG15) was a tumor suppressor which inhibited TMZ resistance through altering tumor microenvironment [28]. It has been reported that NEAT1 was up-regulated and promoted tumor progression in glioma [29], indicating NEAT1 acted as an oncogene in GBM progression. In addition, a study focused on the chemoresistance triple-negative breast cancer (TNBC) revealed that down-regulating NEAT1 enhanced the sensitized cells to chemotherapy and reduced CD44^+^/CD24^−^, ALDH^+^, and SOX2^+^ cell populations, implicating that NEAT1 was closely related to cancer stemness and chemoresistance in TNBC [30]. However, the effects of NEAT1 in TMZ resistance in GSCs remain to be illustrated. In the present study, we identified GSCs had lower sensitivity to TMZ and higher expression of NEAT1, compared with non-GSCs. We also found NEAT1 knockdown further impaired the proliferation, migration and invasion phenotypes of GSCs induced by TMZ treatment, indicating that knockdown NEAT1 decreased the resistance of GSCs to TMZ.

MiRNAs usually negatively regulate gene expression post-transcriptionally by binding to the 3′-UTR of target mRNA [31]. miRNAs are engaged in the regulation of multiple cellular behaviors such as growth, proliferation, survival and death in pathological conditions including cancer [32]. A large amounts of researches have suggested that miRNAs are related to TMZ resistance in GBM, including miR-195, miR-9 and miR-125b [33–35]. Previous study showed that let-7g-5p was significantly downregulated in GBM patients, and overexpressing let-7g-5p inhibited epithelial–mesenchymal transition (EMT) phenotypes and stem cell phenotypes and TMZ resistance by targeting V-set and immunoglobulin domain containing 4 (VSIG4) [23]. Here, we performed gain of function and studied the effects on the malignant behaviors of GSCs. Results showed that overexpression of let-7g-5p suppressed the proliferation, migration and invasion phenotypes of GSCs on the basis of TMZ treatment, implying let-7g-5p up-regulation reduced the TMZ resistance of GSCs. Moreover, we also found that let-7g-5p could interact with NEAT1 and negatively affected the biological roles mediated by NEAT1 in GSCs, indicating that let-7g-5p was one of the function targets of NEAT1-mediated TMZ resistance of GSCs.

Mitogen-activated protein kinases (MAPKs) are evolutionarily conserved proteins which work as a critical regulator in a variety of cellular physiologies [9]. A great number of reports have confirmed that the activation of MAPKs was positively correlated to GBM progression and TMZ resistance [36–38]. For instance, the activation of p38 MAPK pathway elevated the expression of Nrf2, and eventually increasing the sensitivity of glioma cells to TMZ [38]. MAP3K1 was a key isoform for the first stimulation step of MAPKs and worked as an oncogene involved in the regulation of cell growth, migration, apoptosis and chemoresistance in multiple cancers such as gastric cancer, glioma, breast cancer [9,39,40]. Wang et al. reported an elevated MAP3K1 expression in glioma, which was negatively associated with a poor prognosis, and could promote the sensibility of GBM cell to TMZ and radiotherapy by combining with TRIB2 [9]. These observations have implied that MAP3K1 may be a regulator of chemoresistance and tumor development. Here, the enriched MAP3K1 expression in GBM patients was found, and it was directly bound by let-7g-5p, thus positively regulated by NEAT1. Furthermore, MAP3K1 overexpression restored NEAT1-induced impairment of malignant behaviors and TMZ resistance of GSCs, suggesting that MAP3K1 was a downstream functional target of NEAT1/let-7g-5p axis mediated TMZ resistance of GSCs.

In summary, we proposed that a mechanism of action mediated by NEAT1 on the phenotypes and TMZ resistance of GSCs, that is, NEAT1 down-regulation reduced the TMZ resistance and malignant phenotypes of GSCs by regulating let-7g-5p/MAP3K1 axis, and eventually delaying the progression of GBM. Therefore, therapies that target the NEAT1/let-7g-5p/MAP3K1 axis may provide some useful insight into solving TMZ resistance of GBM.

## Abbreviations

bFGF: basic fibroblast growth factor
BSA: bovine serum albumin
CCK-8: Cell Counting Kit-8
DMEM: Dulbecco’s Modified Eagle’s Medium
DMEM/F12: Dulbecco's modified Eagle's medium and Ham's F12
EGF: epidermal growth factor
EMT: epithelial–mesenchymal transition
FBS: fetal bovine serum
FcR: Fc receptor
GB: glioblastoma
GBM: glioblastoma multiforme
GSC: glioma stem cell
HEK: human embryonic kidney
lncRNA: long non-coding RNA
MAPK: mitogen-activated protein kinase
MAP3K1: mitogen-activated protein kinase kinase kinase 1
miRNA: microRNA
MUT: mutant type
NC: negative control
NEAT1: nuclear enriched abundant transcript 1
PBS: phosphate-buffered saline
qRT-PCR: quantitative real-time PCR
shRNA: short hairpin RNA
SNHG15: small nucleolar RNA host gene 15
SOX9: SRY-box transcription factor 9
TBST: Tris Buffered Saline Tween
TMZ: temozolomide
TNBC: triple-negative breast cancer
VSIG4: V-set and immunoglobulin domain containing 4
WT: wild-type
3′-UTR: 3′-untranslated region
